# Oncogenic transformation of human lung bronchial epithelial cells induced by arsenic involves ROS-dependent activation of STAT3-miR-21-PDCD4 mechanism

This article has been retracted.

**DOI:** 10.1038/srep37227

**Published:** 2016-11-23

**Authors:** Poyil Pratheeshkumar, Young-Ok Son, Sasidharan Padmaja Divya, Lei Wang, Zhuo Zhang, Xianglin Shi

**Affiliations:** 1 Center for Research on Environmental Disease, University of Kentucky, 1095 VA Drive, Lexington, KY 40536, USA; 2 Department of Toxicology and Cancer Biology, University of Kentucky, 1095 VA Drive, Lexington, KY 40536, USA

## Abstract

Arsenic is a well-documented human carcinogen. The present study explored the role of the onco-miR, miR-21 and its target protein, programmed cell death 4 (PDCD4) in arsenic induced malignant cell transformation and tumorigenesis. Our results showed that treatment of human bronchial epithelial (BEAS-2B) cells with arsenic induces ROS through p47^phox^, one of the NOX subunits that is the key source of arsenic-induced ROS. Arsenic exposure induced an upregulation of miR-21 expression associated with inhibition of PDCD4, and caused malignant cell transformation and tumorigenesis of BEAS-2B cells. Indispensably, STAT3 transcriptional activation by IL-6 is crucial for the arsenic induced miR-21 increase. Upregulated miR-21 levels and suppressed PDCD4 expression was also observed in xenograft tumors generated with chronic arsenic exposed BEAS-2B cells. Stable shut down of miR-21, p47^phox^ or STAT3 and overexpression of PDCD4 or catalase in BEAS-2B cells markedly inhibited the arsenic induced malignant transformation and tumorigenesis. Similarly, silencing of miR-21 or STAT3 and forced expression of PDCD4 in arsenic transformed cells (AsT) also inhibited cell proliferation and tumorigenesis. Furthermore, arsenic suppressed the downstream protein E-cadherin expression and induced β-catenin/TCF-dependent transcription of uPAR and c-Myc. These results indicate that the ROS-STAT3-miR-21-PDCD4 signaling axis plays an important role in arsenic -induced carcinogenesis.

Arsenic has been classified as a class I human carcinogen for lung cancer by the International Agency of Research on Cancer^1^. Long-term exposure to arsenic in drinking water is increasingly recognized as a major public health concern in several regions of the world^2^,^3^. Generation of reactive oxygen species (ROS) has been described as one of the earliest and most important mechanisms of arsenic-induced carcinogenicity^4^,^5^,^6^,^7^,^8^,^9^. Studies also point the role of epigenetic mechanisms in arsenic induced malignant transformation and tumorigenesis; changes may include DNA methylation patterns, histone modification and altered expression of microRNAs (miRNAs)^10^.

MicroRNAs are a class of endogenous RNA molecules 19–25 nucleotides in length that are able to regulate genes at the post-transcriptional level by binding to the target 3′ untranslated region (UTR), and promote target gene cleavage or translational inhibition^11^. Growing evidence shows that miRNAs play an important role in metal carcinogenesis^12^. Among them, miR-21 has emerged as a key oncomir, since it is upregulated in a wide range of cancers^13^,^14^,^15^,^16^, and implicated in multiple malignancy-related processes such as cell proliferation, apoptosis, invasion, and metastasis^17^,^18^,^19^. Functional studies show that knockdown of miR-21 leds to reduced proliferation and tumor growth in MCF- 7 cells^20^,^21^, and reduced invasion and metastasis in MDAMB-231 cells^21^. A recent study suggests that NADPH oxidase (NOX)-derived ROS is essential for the expression and function of miR-21 22.

Previous studies demonstrated that miR-21 post-transcriptionally down-regulates the tumor suppressor PDCD4 23,24, which has been implicated in the development and progression of several human cancers^25^,^26^,^27^,^28^,^29^. PDCD4 knockdown stimulated the invasion of colon tumor HT29 cells and inhibited E-cadherin expression with an accumulation of active β-catenin in the nuclei, and associated stimulation of β-catenin/T cell factor (TCF)-dependent transcription of genes such as uPAR and c-Myc^30^,^31^. Constitutive activation of the signal transducer and activator of transcription-3 (STAT-3) is detected in many human cancers^32^,^33^,^34^ and has been implicated in tumor cell survival, proliferation, invasion, and angiogenesis^35^. Reports indicate that inhibition of phospho-STAT3 led to a decrease in miR-21 expression, and an increase in PDCD4 expression as well as the migration and invasion of hepatocellular carcinoma cells^36^. However, the mechanisms by which miR-21 acts in the development of arsenic-induced carcinogenesis remain unknown.

For the first time, the present study explores the role of the STAT3-miR-21-PDCD4 signaling cascade in arsenic-induced malignant cell transformation. We found that chronic arsenic exposure increased miR-21 levels and was associated with inhibition of PDCD4 expression and malignant cell transformation. Importantly, arsenic-induced ROS was essential for the miR-21 increase and PDCD4 reduction. In addition, STAT3 transcriptional activation by IL-6 was crucial for the arsenic-induced miR-21 increase. Furthermore, silencing of miR-21 or STAT3 and overexpression of PDCD4 or catalase in BEAS-2B cells reduced malignant transformation and tumorigenicity in nude mice after chronic arsenic exposure. These results suggest that malignant transformation of human lung bronchial epithelial cells induced by arsenic involves a ROS-dependent activation of a STAT3-miR-21-PDCD4 system.

## Results

### Arsenic increases ROS generation

Arsenic -induced ROS production was quantified by flow cytometry using the fluorescent probes DHE and DCFDA. Arsenic exposure dramatically stimulated O_2_^.−^ and H_2_O_2_ generation in BEAS-2B cells, as indicated by an increase of DHE (Fig. 1A) and DCFDA (Fig. 1B) fluorescence intensity, respectively, when levels were compared to those generated from untreated control cells. Our previous studies show that pretreatment with MnTMPyP decreased O_2_^.−^ generation and catalase decreased H_2_O_2_ production, respectively induced by arsenic^37^. Furthermore, the arsenic-induced ^•^OH generation in BEAS-2B cells was detected by Electron spin resonance (ESR) (Fig. 1C). NOX activity was significantly (p < 0.05) increased in arsenic-treated cells within 6 h and the effect lasted up to 24 h (Fig. 1D). Moreover we found that acute arsenic treatment also increased the expression of p47phox, one of the NOX subunits (Fig. 1E). Previous studies from our group showed that pretreatment with apocynin (NOX inhibitor) decreased arsenic-induced O_2_^.−^ and H_2_O_2_ generation in BEAS-2B cells^37^. Taken together, these results suggest that arsenic exposure induces ROS production in BEAS-2B cells, and that activation of NOX is required for this ROS generation.

### Arsenic increases miR-21 and targets PDCD4

Studies have shown that PDCD4 is an important functional target of the oncomiR, miR-21 23. In this study, we observed a dose-dependent and significant (p < 0.05) increase in miR-21 levels, associated with a decrease in PDCD4 expression in BEAS-2B cells treated with arsenic using RT-PCR and Western blot analysis respectively (Fig. 1F,G). Similar results for PDCD4 were observed by immunofluorescence with diminished PDCD4 expression in the nucleus after acute arsenic treatment (Fig. 1H). There was a significant decrease in the PDCD4 3′-UTR reporter activity when cells were treated with 10 μM arsenic for 6 h, whereas reporter activity was upregulated when miR-21 gene expression was inhibited (Fig. 1I). These results support the assumption that acute arsenic treatment increases the miR-21 levels with an associated decrease in PDCD4 expression.

Next we studied the role of arsenic-induced ROS generation in miR-21- PDCD4 signaling. We demonstrated that exogenous addition of ROS inhibitors, NAC or Catalase markedly ameliorates the arsenic-induced miR-21 elevation and PDCD4 suppression in BEAS-2B cells using RT-PCR and Western blot analysis respectively (Figs. 1J,K). These results provide solid evidence that ROS plays a key role in arsenic-induced miR-21 elevation and PDCD4 reduction.

### miR-21 induction by arsenic is strictly STAT3 dependent

STAT3 binding to the miR-21 promoter upon IL-6 induction has been reported previously^38^. A genomic DNA fragment extending from −1120 to +25 bp relative to the miR-21 transcription start site containing the putative STAT3 enhancer region proved to be IL-6–responsive in a reporter assay^38^. To investigate whether, arsenic induces an IL-6 mediated STAT3 binding to the miR-21 promoter, we analyzed IL-6 levels and STAT3 activation by ELISA, and STAT3 binding to the miR-21 promoter by ChIP assay. Acute arsenic treatment to BEAS-2B cells significantly (p < 0.05) increased the IL-6 levels (Fig. 2A), STAT3 transcriptional activation (Fig. 2B), and STAT3 phosphorylation (Fig. 2C) in a dose-dependent manner. The role of ROS in IL-6 induction and STAT3 activation was verified by the addition of H_2_O_2_ (Fig. 2A,B). STAT3 phosphorylation by arsenic was confirmed by immunofluorescence staining (Fig. 2D). As shown in Fig. 2E, miR-21 promoter activity was significantly (p < 0.05) increased by arsenic and IL-6, while STAT3 knock down (siSTAT3) inhibited miR-21 promoter activities relative to their respective vector controls. Moreover, both arsenic and IL-6 treatments increased the binding of STAT3 on the miR-21 promoter (Fig. 2F-G).

### Activation of the STAT3-miR-21-PDCD4 signaling axis contributes to arsenic induced malignant cell transformation

Malignant cell transformation was assessed by anchorage-independent growth in soft agar^39^. BEAS-2B cells were treated with selected concentrations (0.125, 0.25 and 0.5 μM) of arsenic for six months. Chronic exposure (6 months) to low concentrations of arsenic (0.1, 0.25 and 0.5 μM) induced malignant transformation of BEAS-2B cells as shown by the marked increase in size and number of colonies compared to untreated control (Fig. 3A,B). The chronic treatment of arsenic significantly (p < 0.05) increased miR-21 levels in a time and dose dependent manner (Fig. 3C). We also found a dose-dependent and drastic decrease in the PDCD4 expression and increase in the p47phox expression and STAT3 phosphorylation with chronic arsenic exposure (Fig. 3D). Similar results were observed by immunofluorescence; BEAS-2B cells treated with arsenic (0.5 μM) for six months showed a marked decrease in the PDCD4 level and increase in the STAT3 phosphorylation (Fig. 3E). The above results demonstrate a role for miR-21-PDCD4 signaling in arsenic-induced transformation.

### Arsenic-induced ROS generation and STAT3 activation is essential for miR-21 increase and PDCD4 suppression

To determine whether ROS plays an important role in chronic arsenic-induced miR-21 increase and PDCD4 suppression, catalase was overexpressed in BEAS-2B cells (Fig. 4A) and treated with arsenic (0.5 μM) for six months. Forced expression of catalase markedly inhibited miR-21 expression (Fig. 4B) and suppressed the PDCD4 reduction (Fig. 4C) induced by chronic arsenic treatment. Importantly, catalase overexpression also decreased the chronic arsenic-induced malignant cell transformation (Fig. 4D). Knockdown of p47phox in BEAS-2B cells (Fig. 4E) noticeably decreased the arsenic-induced increase in miR-21 expression (Fig. 4F) and suppressed the PDCD4 reduction (Fig. 4G). Interestingly, silencing p47phox significantly inhibited chronic arsenic-induced oncogenic transformation (Fig. 4H). These results clearly demonstrate the indispensable role of ROS in regulating miR-21-PDCD4 signaling during chronic arsenic-induced malignant cell transformation.

To verify the crucial role of STAT3 activation in arsenic-induced miR-21 increase, PDCD4 suppression and malignant transformation, STAT3 expression was stably silenced in BEAS-2B cells (shSTAT3) and treated with arsenic (0.5 μM) for six months. Silencing of STAT3 in BEAS-2B cells dramatically decreased the arsenic-induced increase in miR-21 expression (Fig. 4I), and suppressed the PDCD4 reduction (Fig. 4J) and subsequent malignant transformation (Fig. 4K).

### Silencing of miR-21 and forced expression of PDCD4 inhibit arsenic-induced oncogenic transformation

To investigate the oncogenic role of miR-21 in arsenic-induced malignant transformation, BEAS-2B cells with stable knock down of miR-21 were treated with arsenic (0.5 μM) for six months. Figure 5A shows that cells with miR-21 knock down exhibited no increase in miR-21 levels even after chronic arsenic treatment. Knock down of miR-21 in BEAS-2B cells markedly inhibited the chronic arsenic-induced PDCD4 suppression (Fig. 5B). Importantly, miR-21 knock down significantly (p < 0.05) reduced the chronic arsenic-induced malignant cell transformation (Fig. 5C). As expected, forced expression of PDCD4 in BEAS-2B cells (Fig. 5D) significantly (p < 0.05) decreased the chronic arsenic-induced malignant cell transformation (Fig. 5E). The above results clearly indicate that increased levels of the oncomiR miR-21 and suppression of tumor suppressor PDCD4 are critically important for arsenic-induced malignant cell transformation.

### Upregulation of miR-21 and suppression of PDCD4 by chronic arsenic exposure induces tumorigenesis of BEAS-2B cells *in vivo*

Next we investigated whether the increase in miR-21 levels and PDCD4 suppression mediated by chronic arsenic exposure in BEAS-2B cells induces tumors in nude mice. Nude mice were injected sc with BEAS-2B cells that had been exposed to arsenic for 6 months at the indicated concentration. Over a 4-week period post inoculation, we observed visible tumor formation that increased progressively in size for mice injected with arsenic-treated BEAS-2B cells but not in those injected with control cells (Fig. 6A,B). Consistent with our *in vitro* findings above, we found significantly increased miR-21 levels (Fig. 6C) associated with decreased PDCD4 expression (Fig. 6D,E) and increased phosphorylated STAT3 (Fig. 6F) in xenograft tumors generated with chronic arsenic exposed BEAS-2B cells.

In addition, we demonstrated that stable knockdown of miR-21 and STAT3, or overexpression of PDCD4 or catalase in BEAS-2B cells that had been chronically exposed to arsenic reduced tumorigenicity in nude mice. For these studies, BEAS-2B cells stably silenced with shRNA’s for miR-21 or STAT3, or transfected with plasmids overexpressing catalase or PDCD4, were exposed to arsenic for 6-months. Treated cells were injected into nude mice and tumor development was assessed four weeks post-injection. Tumors developed from arsenic-exposed BEAS-2B cells with stable knockdown of miR-21 or STAT3, and tumors formed from arsenic-exposed BEAS-2B cells overexpressing PDCD4 or catalase were smaller than those from the corresponding vector cells exposed to arsenic (Fig. 7A,B). Moreover, tumors developed from arsenic-exposed BEAS-2B cells with stable knockdown of miR-21 or STAT3, and tumors formed from arsenic-exposed BEAS-2B cells overexpressing PDCD4 or catalase showed a decreased miR-21 levels (Fig. 7C) and increased PDCD4 expressions (Fig. 7D) compared to those tumors developed from the corresponding-vector cells exposed to arsenic.

### Stable knockdown of miR-21 or STAT3 and overexpression of PDCD4 in AsT cells suppresses tumorigenesis

The arsenic-transformed cells (AsT) from anchorage-independent colonies were selected and grown in DMEM (Fig. 8A). Passage-matched cells without arsenic treatment were used as the control. Increased miR-21 levels (Fig. 8B) and decreased PDCD4 expression (Fig. 8C) in AsT cells compared to passage-matched cells was observed. The clonogenic assay (Fig. 8D,E) showed that AsT cells formed more colonies compared to passage-match cells, and that knockdown of miR-21 or STAT3 and that overexpression of PDCD4 in AsT cells significantly (p < 0.05) reduced the colony number. (**F–J**) We observed a visible tumor formation that progressively increased in size in mice injected with AsT cells compared to passage-match cells, while the tumors were small from mice injected with AsT cells stably knockdown with miR-21 or STAT3 and overexpressing of PDCD4 (Fig. 8F,G). Furthermore, tumors developed from AsT cells with stable knockdown of miR-21 or STAT3 and those overexpressing PDCD4 showed decreased miR-21 levels (Fig. 8H), increased PDCD4 expression (Fig. 8I) and decreased levels of phosphorylated STAT3 (Fig. 8J) compared to those tumors developed from AsT-vector cells.

### PDCD4 suppression by arsenic down-regulates E-cadherin and stimulates β-catenin/TCF-dependent transcription of uPAR and c-Myc

Previous studies reported that suppression of PDCD4 elicits an inhibition of E-cadherin expression, which is associated with an increase in β- catenin activation and TCF4 expression^31^. To confirm this in our model system, BEAS-2B cells were exposed to various doses of arsenic for a short (24 h) or extended (6 mo) time period. Results show that both acute (Fig. 9A) and chronic (Fig. 9B) arsenic treatment of BEAS-2B cells down-regulated E-cadherin protein expression with an associated up-regulation of active β-catenin (nuclear translocated form) and TCF4, whereas the level of total β-catenin remained unchanged. Immunofluorescence staining confirmed that chronic arsenic exposure decreased E-cadherin expression (Fig. 9C) and increased β- catenin (Fig. 9D) and TCF4 accumulation in the nucleus (Fig. 9E). These data clearly show that arsenic exposure suppresses E-cadherin and increases the accumulation of β- catenin and TCF4 in the nucleus during malignant transformation.

Reports indicate that uPAR and c-Myc are the target genes of β-catenin/TCF4 dependent transcription^31^. The c-Myc oncogene plays vital roles for both early and late stages of carcinogenesis^40^. uPAR is involved in cancer cell invasion and significantly correlates to tumor aggressiveness and poor outcome^41^. Chronic arsenic exposure increased c-Myc and uPAR expressions in BEAS-2B cells in a dose-dependent manner (Fig. 10A). Similarly, the invasive potential of BEAS-2B cells under chronic arsenic exposure was also increased in association with uPAR expression (Fig. 10B,C). BEAS-2B cells treated with arsenic (0.5 μM) for 6 months showed a 5-fold increase in invasive potential compared to untreated control cells (Fig. 10C). A previous study demonstrated that in cells with PDCD4 knock down, β-catenin binds with TCF4 in the nucleus, with subsequent binding this complex to the uPAR and c-Myc promoters^31^. To investigate this as a potential mechanism for arsenic-induced carcinogenesis, we performed ChIP analysis using a TCF4 antibody and primers that specifically amplify the β-catenin/TCF4 binding site on the promoters of uPAR (−308 to −302) and c-Myc (−452 to −446). As shown in Fig. 10D,E, association of the β-catenin/TCF4 complex to the uPAR and c-Myc promoters increased during chronic arsenic treatment in a dose-dependent manner. These results indicate that PDCD4 suppression increases uPAR and c-Myc expressions, and also activates β-catenin/TCF4 complex binding to the uPAR and c-Myc promoters during chronic arsenic exposure.

## Discussion

Arsenic induces human cancers including lung cancer^42^ and can affect the expression of certain miRNAs^43^,^44^. Increasing evidence indicates that abnormal expression of miRNAs is associated with carcinogenesis^45^. miR-21 is a key oncogene, plays an important role in the initiation and progression of cancer^46^ and is highly overexpressed in most cancers^47^,^48^,^49^. miR-21 binds to the 3′-UTR of PDCD4 and suppresses its translation^24^. Inhibition of miR-21 or overexpression of PDCD4 results in decreased tumor formation and growth^50^. Therefore, miR-21 and PDCD4 are potential novel targets for cancer prevention or for cancer therapeutics. In this study, we focused on the functions and regulatory mechanisms of miR-21 in arsenic induced cellular transformation, invasion and tumorigenesis by directly targeting the tumor suppressor PDCD4.

We previously reported that the miR-21 was significantly upregulated, with an associated inhibition of PDCD4 expression, in different lung cancer cells (H2030, H460, H23, and A549) compared to normal lung epithelial cells (BEAS-2B and NL-20)^51^. In the current study, arsenic treatment robustly increased miR-21 levels with an associated decrease in PDCD4 expression in BEAS-2B cells. These results, verified by immunofluorescence analysis of PDCD4, showed that arsenic treatment reduced PDCD4 expression in the nucleus. Similar results were observed in lung^52^, colon^53^, prostate^53^, ovarian^28^ and oral cancers^54^. In these cancers, loss of PDCD4 expression was associated with disease progression. Furthermore, arsenic treatment also decreased PDCD4 3′-UTR reporter activity. Upregulation of miR-21 and inhibition of PDCD4 by chronic arsenic treatment induced malignant transformation and tumorigenesis of BEAS-2B cells. Stable shut down of miR-21 and overexpression of PDCD4 in BEAS-2B cells significantly inhibited the arsenic induced malignant transformation and tumorigenesis. As expected, elevated miR-21 and inhibition of PDCD4 expression was observed in arsenic transformed (AsT) cells. Knockdown of miR-21 and overexpression of PDCD4 in AsT cells also inhibited cell proliferation and tumorigenesis. These results strongly indicate that miR-21-PDCD4 signaling plays an important role in arsenic induced malignant transformation and tumorigenesis.

It has been established that arsenic-induced ROS is vital for malignant cell transformation^37^. Hydrogen peroxide (H_2_O_2_) upregulates miR-21 and decreases PDCD4 expression in vascular smooth muscle cells^55^. However, the role of arsenic -induced ROS on miR-21-regulated malignant transformation in BEAS2B cells remains unclear. In this study, we found that arsenic induces ROS and p47^phox^ expression; p47^phox^ is a NOX subunits and is the key source of arsenic-induced ROS. Interestingly, stable knockdown of p47^phox^ and overexpression of catalase in BEAS-2B cells markedly suppressed the arsenic-induced miR-21 up-regulation and PDCD4 inhibition, and thereby prevented malignant transformation and tumorigenesis. These results clearly point to arsenic-induced ROS production as an essential event in the activation of the miR-21-PDCD4 signaling axis and subsequent malignant transformation.

We also investigated the role of miR-21 regulation in cell transformation and tumorigenesis. Following IL-6 induction, STAT3 reportedly binds directly to the miR-21 promoter, which promotes cancer cell survival and proliferation^38^,^56^,^57^. In this study, we showed that arsenic treatment increases the IL-6 levels, STAT3 transcriptional activation, and STAT3 phosphorylation in BEAS-2B cells. In addition, the binding affinity of STAT3 on miR-21 promoter was also increased during arsenic exposure. The role ROS in the induction of IL-6 and STAT3 activation was verified by the addition of H_2_O_2_. Stable knockdown of STAT3 markedly decreased arsenic-induced miR-21 upregulation and malignant transformation. Similar results were observed in hepatocellular carcinoma cells, where STAT3 inhibition decreased the miR-21 upregulation^36^. Furthermore, silencing STAT3 also decreased AsT cells proliferation and tumorigenesis. From these results, we infer that arsenic-induced IL-6 mediates STAT3 activation, which is crucial for miR-21 upregulation during lung carcinogenesis.

It has been already reported that downregulation of PDCD4 leads to the inhibition of E-cadherin expression, with an associated increase in β-catenin/TCF4 dependent transcription^31^. The current study demonstrates that both acute and chronic treatment of arsenic suppressed the E-cadherin expression with an associated increase in active β-catenin and TCF4 expression in BEAS-2B cells in a dose-dependent manner. In addition, chronic arsenic exposure increased uPAR and c-Myc protein expressions in BEAS-2B cells as well as cellular invasive potential. Furthermore, chronic arsenic exposure increased the binding of TCF4 on uPAR and c-Myc promoters. These findings indicate that PDCD4 suppression is critical for β-catenin/TCF dependent transcription of c-Myc, and uPAR during arsenic induced lung carcinogenesis.

In summary, we found that chronic arsenic exposure to BEAS-2B cells increases miR-21 levels with an associated inhibition of PDCD4 expression, and causes malignant transformation and tumorigenesis (Fig. 10F). Arsenic elicits an upregulation in miR-21 via the IL-6/STAT3 pathway. Importantly, arsenic-induced ROS is essential for the activation of the STAT3-miR-21-PDCD4 signaling axis. Overall, our findings demonstrate an active involvement of a ROS-STAT3-miR-21-PDCD4 signaling axis in arsenic-induced malignant cell transformation and tumorigenesis.

## Materials and Methods

### Antibodies and chemicals

Sodium arsenite (NaAsO_2_) and 5,5-dimethyl-1-pyrroline-1-oxide (DMPO), were purchased from Sigma-Aldrich (St Louis, MO). Both Dichlorodihydrofluoresceine acetate (DCFDA) and dihydroethidium (DHE) were from Molecular Probes (Eugene, OR). Human miR-21 hairpin inhibitor was purchased from Thermo Fisher Scientific Dharmacon (Chicago, IL, USA). Antibodies against PDCD4 (CST#9535), E-cadherin (CST#3195), β-catenin (CST#8480), c-Myc (CST#5605), uPAR (CST#9692), pSTAT3 Tyr705 (CST#9145) and STAT3 (CST#9139) were purchased from Cell Signaling Technology (Danvers, MA). Anti–active-β-catenin (clone 8E7#05-665) antibody was purchased from EMD Millipore (Billerica, MA). Antibodies against TCF4 (sc-13027) and GAPDH (sc-25778) were purchased from Santa Cruz Biotechnology, Inc. (Santa Cruz, CA).

### Cell lines and cell culture

The human bronchial epithelial cell line BEAS-2B was obtained from the American Type Culture Collection (Rockville, MD). Arsenic transformed cells (AsT) were generated as described previously^58^. BEAS-2B and AsT cells were cultured in Dulbecco’s modified Eagle’s medium (DMEM) supplemented with 10% fetal bovine serum (FBS), 2mM L-glutamine, and 5% penicillin/streptomycin at 37 °C in a humidified atmosphere with 5% CO_2_ in air.

### Plasmids and Transfection

Plasmid DNA encoding human catalase and STAT3 shRNA was purchased from Origene (Rockville, MD). PDCD4 3′-UTR reporter plasmid was kindly provided by Dr. Yong Li (University of Louisville, USA). The STAT3-miR-21 reporter was constructed as described previously^38^. PcDNA3.1/PDCD4 plasmid was kindly provided by Dr. Hsin-Sheng Yang (University of Kentucky, USA). The miR-21 shRNA was purchased from Applied Biological Materials, Inc. (Richmond, CA). Protocols for the overexpression of catalase and PDCD4 and knockdown of STAT3, miR-21 in BEAS-2B cells and generation of AsT have been described previously^51^. The stable silencing of p47phox in BEAS-2B cells was performed as described previously^59^.

### Intracellular ROS determination

Generation of H_2_O_2_ and O_2_^**−**^ was assessed using the fluorescent dye DCFDA and DHE, respectively, as described previously^60^. The cells were cultured in 6-well plates (2 × 10^5^ cells/well), treated with arsenic for 12 h and incubated with DCFDA or DHE (10 μM) for 40 min at 37 °C. Trypsinized cells were washed twice with cold phosphate buffered saline (PBS), and analyzed by fluorescence-activated cell sorting (FACS Calibur, BD Biosciences). The fluorescence intensity of DCFDA was measured with an excitation at 492 nm and emission at 517 nm. The fluorescence intensity of DHE was measured with an excitation at 535 nm and emission at 610 nm.

### Electron spin resonance (ESR) assay

ESR measurement was conducted using a Bruker EMX spectrometer (Bruker Instruments, Billerica, MA) and a flat cell assembly. The intensity of ESR signal determined the amount of hydroxyl radical generated. DMPO, used as a spin or radical trap, was charcoal purified and distilled to remove all ESR detectable impurities before use. Hyperfine couplings were measured (to 0.1 G) directly from magnetic field separation using potassium tetraperoxochromate (K_3_CrO_8_) and 1,1-diphenyl-2-picrylhydrazyl (DPPH) as reference standards. Reactants were mixed in test tubes to a total final volume of 0.5 mL. The reaction mixture was then transferred to a flat cell for ESR measurement.

### NOX activity assay

NOX activity was measured by the lucigenin enhanced chemiluminescence method as described^59^. Briefly, cultured cells were homogenized in lysis buffer followed by centrifugation to remove the unbroken cells and debris. 100 μL of homogenates were added to 900 μL of 50 mM phosphate buffer. Relative light units of photon emission were measured in Glomax luminometer (Promega).

### Luciferase reporter assay

BEAS-2B cells transfected with the luciferase reporter constructs were seeded into 24-well plates (5 × 10^4^/well) grown to 80–90% confluence and treated as indicated. Cellular lysates were subjected to a luciferase reporter assay (Promega) using the Glomax luminometer as described previously^60^. The results are expressed as relative activity normalized to the luciferase activity in the control cells without treatment.

### ELISA for IL-6 and STAT3

BEAS-2B cells were cultured in DMEM supplemented with 10% FBS containing arsenic (0, 5, and 10 μM) for 24 h. Subsequently, the culture media was collected and used to estimate IL-6 level using a commercially available IL-6 ELISA kit (BioLegend, Inc. CA, USA) according to the manufacturers’ instructions. For quantitative analysis of STAT3, Trans^AM^ ELISA kit (Active Motif, Carlsbad, CA) was used following the manufacturer’s protocol. For this assay, the nuclear extracts of cell samples from various treatment groups were prepared using the Nuclear Extraction kit (Active Motif) according to the manufacturer’s instructions. Absorbance was recorded at 450 nm with reference taken at 650 nm. The assay was performed in duplicate and the results are expressed as a percentage, relative to the absorbance for the control group.

### Arsenic-induced cell transformation and anchorage-independent colony growth

Soft agar colony formation was performed as described previously^60^. BEAS-2B cells, or BEAS-2B cells with stable overexpression of catalase or PDCD4, or BEAS-2B cells with stable knockdown of p47phox, STAT3 or miR-21, were treated with 0.5 μM arsenic. Medium was replaced every 3 days. After 24 weeks, 1 × 10^4^ cells were suspended in 3 mL culture medium containing 0.35% agar and seeded onto 6-well plates with a 0.5% agar base layer, and maintained in an incubator for 4 weeks. Colonies greater than 0.1 mm in diameter were scored by microscopic examination. Arsenic-transformed cells from anchorage-independent colonies were selected and grown in DMEM and passage-matched cells with no arsenic treatment were used as the control.

### Chromatin immunoprecipitation (ChIP) assay

ChIP analysis was performed using a PierceTM Agarose ChIP Kit (Thermo Scientific, Rockford, IL). Sheared chromatin was diluted and immunoprecipitated with 2 μg of anti-STAT3, anti-TCF4 or control IgG antibody. DNA protein complexes were eluted from protein A/G agarose beads using a spin column and were reverse cross-linked by incubating with NaCl at 65 °C. The relative TCF4 binding to the c-MYC and uPAR promoters or STAT3 binding to miR-21 promoter was analyzed by MyiQ™ Single-Color Real-Time PCR Detection System (Bio-Rad, Hercules, CA) with SYBR Green PCR master mix using following primer sequences, STAT3 binding to miR-21 promoter/enhancer (F) CCTCTGAGAAGAGGGGACAA and (R) ACCGCTTCCAGCAAAAGAGT. General PCR amplification also performed in a Mastercycler thermal cycler (Eppendorf, Foster City, CA).

### Quantitative real-time polymerase chain reaction (qRT-PCR)

Total RNA was extracted using Trizol (Invitrogen), and cDNA was synthesized by using TaqMan microRNA reverse transcriptase kit (Applied Biosystems, Foster City, CA, USA) according to the manufacturer recommendations. Expression of miR-21-microRNA was determined by the TaqMan miRNA-assay (Applied Biosystems), and normalized using the 2^−ΔΔCT^ -method relative to U6-snRNA. All TaqMan-PCR reactions were performed in triplicate using a Bio-Rad’s MyiQTM single-color real-time PCR detection system.

### Western blot analyses

Cell lysates were prepared in RIPA buffer. Lysate protein concentration was measured using Bradford Protein Assay Reagent (Bio-Rad). 30 μg of protein was separated by SDS–PAGE, the proteins transferred to membranes that were incubated with primary antibodies, as indicated. The blots were then re-probed with secondary antibodies conjugated to horseradish peroxidase. Immunoreactive bands were detected by the enhanced chemiluminescence reagent (Amersham, Pittsburgh, PA).

Tumor tissues were homogenized with MagNA Lyser Green Beads using MagNA Lyser Instrument (Roche, Indianapolis, IN) and western blot analysis performed as outlined above.

### Tumorigenesis studies

The animal studies were conducted in accordance with NIH animal use guidelines and the experimental protocol approved by the Institutional Animal Care and Use Committee (IACUC) of the University of Kentucky at Lexington. Athymic nude mice (NU/NU, 6–8 weeks old; Charles River) were housed in a pathogen-free room in the animal facilities at the Chandler Medical Center, University of Kentucky. Cells (2 × 10^6^ cells per mouse) from different treatments were re-suspended in serum-free medium with basement membrane matrix (BD Biosciences) at a 1:1 ratio (total volume = 100 μl) and subcutaneously injected into the flanks of nude mice. Mice were checked daily for tumor appearance, and tumor volume was measured every 3 days for 30 days. Tumor volume was determined by Vernier caliper, following the formula of *A* × *B*^*2*^ × *0.52*, where A is the longest diameter of tumor and B is the shortest diameter. At the end of the experiment, mice were sacrificed; tumors were excised and snap frozen.

### Immunohistochemical staining

Five-μm thick frozen tumor sections were hydrated in PBS, and non-specific binding sites blocked with 10% horse serum in PBS. Sections were stained using Vectastain ABC Kit according to the manufacturer’s protocol (Vector Laboratories, Burlingame, CA). Briefly, the sections were incubated with rabbit anti-PDCD4 (1:100) or anti-pSTAT3 (1:200) antibody for 2 h at room temperature, washed and then incubated with biotinylated secondary antibody for 45 min followed by incubation with ABC reagent. After washing in PBS, color was developed with DAB solution until the desired staining intensity was achieved. Finally, the sections were counterstained with hematoxylin.

### Immunofluorescence analysis

BEAS-2B cells or BEAS-2B cells chronically exposed to arsenic were grown on coverslips in 6-well plates and treated with arsenic. Cells were fixed with ice-cold 100% methanol followed by permeabilization with 0.2% Triton X-100, blocked with 10% horse serum in PBS solution, and incubated with antibodies to PDCD4 (1:500), pSTAT3 (1:100), E-cadherin (1:100), β-Catenin (1:100), or TCF4 (1:100) in buffer A (1% BSA, 0.1% Triton X-100, 10% horse serum in PBS solution) for 1 h at 37 °C. Cells were then incubated with Alexa Fluor 594 goat anti-rabbit or Alexa Fluor 488 goat anti-rabbit antibody and mounted using DAPI. The cells were visualized using digital confocal microscopy (Confocal Fluorescence Imaging Microscope, Leica TCS-SP5) or Olympus BX53 fluorescence microscope.

### Statistical analysis

Presented values are means ± SD. One-way analysis of variance (ANOVA) was used to determine differences among means, with p < 0.05 considered significant.

## Additional Information

**How to cite this article**: Pratheeshkumar, P. *et al*. Oncogenic transformation of human lung bronchial epithelial cells induced by arsenic involves ROS-dependent activation of STAT3-miR-21-PDCD4 mechanism. *Sci. Rep.* **6**, 37227; doi: 10.1038/srep37227 (2016).

**Publisher's note:** Springer Nature remains neutral with regard to jurisdictional claims in published maps and institutional affiliations.

## Figures and Tables

**Figure 1:** Arsenic increases ROS generation and induces an miR-21-PDCD4 signaling cascade. BEAS-2B cells were exposed to arsenic (0 to 10 μM) for 12 h. Arsenic induced generation of the ROS radicals O_2_^−^ and H_2_O_2_ were identified by DHE (**A**) and DCFDA (**B**) staining, respectively. Upper panels show representative images obtained by fluorescence microscopy and the graphs (lower panels) demonstrate fluorescent intensity determined by flow cytometry. (**C**) Generation of ^•^OH as determined by electron spin resonance. The generation of a 1:2:2:1 quartet ESR signal is shown. (**D**) NOX activity, measured after 6, 12 and 24 h arsenic exposure, utilized the lucigenin chemiluminescence assay. Activity increased in a time- and dose-dependent manner. (**E**) Western blot demonstrates an apparent increase in protein levels of the NOX subunit, p47^phox^ with arsenic exposure. (**F–H**) BEAS-2B cells exposed to increasing concentrations (0–10 μm) of arsenic for 24 h. (**F**) The relative miR-21 level was determined by Taqman real-time PCR. (**G**) Immunoblot analysis of PDCD4 protein levels after acute arsenic treatment. Arsenic induced increases in miR-21 and decreases in PDCD4 levels. (**H**) Representative images of fluorescence immunostaining demonstrate decreased PDCD4 expression with arsenic treatment. Dapi: blue-nuclear; Phalloid: red-cytoplasmic actin; PDCD4, green (**I**) BEAS-2B cells were transfected with the renilla reporter construct (pGL3-PDCD4_3′-UTR), miR-21 inhibitor (100 nM), negative control (100 nM), or pGL3-promoters and treated with 10 μM arsenic for 6 h. Cellular lysates were subjected to a luciferase reporter analysis as described in Materials and Methods and results are expressed as a relative activity (relative luminescence units, (RLU) normalized to the luciferase activity in the vector control cells without treatment. Arsenic increased the binding of miR-21 to the 3′-UTR of PDCD4. Exogenous addition of ROS inhibitors catalase or NAC inhibited the acute arsenic-induced (**J**) miR-21 increase and (**K**) PDCD4 suppression. Data presented in the bar graphs are the mean ± SD of three independent experiments. *Indicates a statistically significant difference from control cells with p < 0.05.

**Figure 2:** Arsenic initiates an IL-6-mediated STAT3 binding to the miR-21 promoter. (**A–C**) BEAS-2B cells were treated with arsenic (5 and 10 μM) for 24 h. (**A**) Increased IL-6 levels in culture medium and (**B**) STAT3 activity in the nuclear fraction of cell lysate were assessed using ELISA kits, following the manufacturer’s protocol. H_2_O_2_ (0.1 mM) and IL-6 (10 ng/ml) were used as positive control. (**C**) Total cell lysates were prepared for western blot analysis using specific antibodies against pSTAT3 and STAT3. Arsenic induced an apparent increase in activated levels in the nucleus. (**D**) Representative images of fluorescence immunostaining confirm presence of nuclear pSTAT3 with arsenic treatment (10** **μM). Dapi: blue-nuclear; Phalloid: red-cytoplasmic actin; pSTAT3, green (**E**) Reporter gene assays were performed in BEAS-2B cells transfected with either a luciferase vector driven by the miR-21 promoter/enhancer alone (−) or in the presence of a vector encoding a small hairpin RNA silencing STAT3 expression (siSTAT3). Knockdown of STAT3 reduced promoter activity. (**F–G**) BEAS-2B cells were exposed to IL-6 or arsenic for 30 minutes and subjected to a chromatin immunoprecipitation (ChIP) analysis using anti-STAT3 or IgG isotype control. Co-immunoprecipitated DNA was amplified by PCR with primers specific for the miR-21 upstream enhancer. Both arsenic and IL-6 increased binding to the mi-R21 promoter. Data presented in the bar graphs are the mean ± SD of three independent experiments. *Indicates a statistically significant difference compared to control with p < 0.05.

**Figure 3:** The arsenic-induced miR-21 increase and PDCD4 suppression contribute to malignant cell transformation. BEAS-2B cells were maintained in a medium containing various concentrations of arsenic (0.1, 0.25 and 0.5 μM) for 6 months. (**A,B**) Cells were cultured in 0.35% soft agar for 5 weeks and number of colonies in the entire dish counted. (**A**) Representative images of control (left panel) and arsenic-treated (right panel) colonies. (**B**) Colony number increased in a dose-dependent manner. (**C**) The relative miR-21 level, determined by Taqman real-time PCR, increased in a time- and dose-dependent manner. (**D**) Total cell lysates were prepared for western blot analysis after 2, 4 and 6 months exposure to arsenic using specific antibodies against PDCD4, p47phox, pSTAT3 and STAT3. Apparent protein levels for PDCD4 decreased and P47phox and pSTAT3 increased in a time- and dose-dependent manner. (**E**) Representative images of fluorescence immunostaining for PDCD4 and pSTAT3 after 2, 4 and 6 months exposure to arsenic, and confirm results from western blot analysis. Data presented in the bar graphs are the mean ± SD of three independent experiments. *Indicates a statistically significant difference compared to control with p < 0.05.

**Figure 4:** Arsenic-induced ROS generation and STAT3 activation are essential for the miR-21 increase and PDCD4 suppression. (**A–D**) BEAS-2B cells with stable overexpression of catalase or their corresponding vehicle vector were exposed to arsenic (0 or 0.5 μM) for 6 months. (**A**) Catalase overexpression was verified by western blot analysis. (**B**) The relative miR-21 level was determined by Taqman real-time PCR and decreased with catalase overexpression. (**C**) Cell lysates were prepared to determine the protein level of PDCD4 by western blot analysis. Apparent PDCD4 levels increased with catalase overexpression. (**D**) Anchorage-independent colony growth, assessed as previously described, decreased with catalase overexpression. (**E–H**) p47phox expression was stably knocked down in BEAS-2B cells and exposed to arsenic (0 or 0.5 μM) for 6 months. **(E**) P47phox knockdown was confirmed by western blot analysis. **(F**) Relative miR-21 level, determined by Taqman real-time PCR was decreased. (**G**) Cell lysates were prepared to evaluate PDCD4 protein levels by western blot analysis. An apparent restoration in PDCD4 levels was observed. (**H**) Anchorage-independent colony growth, assessed as previously described, was also decreased compared with respective vector controls. (**I–K**) BEAS-2B cells with stable knockdown of STAT3 or their corresponding vehicle vector were exposed to arsenic (0 or 0.5 μM) for 6 months. (**I**) The Relative miR-21 level, determined by Taqman real-time PCR, decreased compared with respective vector controls. (**J**) Cell lysates were prepared to determine the protein level of PDCD4 by western blot analysis. Apparent PDCD4 levels increased. (**K**) Anchorage-independent colony growth, assessed as previously described, decreased compared with respective vector controls. Data presented in the bar graphs are the mean ± SD of three independent experiments. *Indicates a statistically significant difference compared to control with p < 0.05.

**Figure 5:** Stable knockdown of miR-21 and overexpression of PDCD4 inhibit arsenic-induced malignant cell transformation. (**A–C**) BEAS-2B cells with stable knockdown of miR-21 or their corresponding vehicle vector were exposed to arsenic (0 or 0.5 μM) for 6 months. (**A**) The relative miR-21 level, determined by Taqman real-time PCR, decreased. (**B**) Cell lysates were prepared to evaluate PDCD4 protein levels by western blot analysis. PDCD4 levels showed an apparent increase. (**C**) Anchorage-independent colony growth was assessed as previously described. (**D–E**) BEAS-2B cells stably overexpressing PDCD4 or their corresponding vehicle vector were exposed with arsenic (0 or 0.5 μM) for 6 months. (**D**) Cell lysates were prepared for western blot analysis and confirm expression of PDCD4 protein. (**E**) Anchorage-independent colony growth, assessed as previously described, demonstrate decreased colony formation when compared with respective vector controls. Data presented in the bar graphs are the mean ± SD of three independent experiments. *Indicates a statistically significant difference compared to control with p < 0.05.

**Figure 6:** Increased miR-21 and suppressed PDCD4 expression by chronic arsenic exposure induces tumorigenesis of BEAS-2B cells *in vivo*. BEAS-2B cells exposed to indicated concentration of arsenic for 6 months were injected sc into nude mice. After 4 weeks, mice were euthanized using CO_2_ and tumor was isolated for further examination. (**A**) Representative images of excised tumors and (**B**) graphic representation of tumor volume demonstrate increased growth with arsenic treatment. (**C**) The relative miR-21 level, determined by Taqman real-time PCR, increased with arsenic treatment. (**D**) Immunohistochemical analysis of PDCD4 protein showed decreased expression with increasing arsenic concentration. (**E**) Protein levels for PDCD4 and pSTAT3, analyzed by western blot, showed an apparent decrease in PDCD4 and apparent increase in pSTAT3 expressions with arsenic exposure. (**F**) Increased STAT3 phosphorylation with arsenic exposure was verified by immunohistochemistry. Data presented in the bar graphs are the mean ± SD of three independent experiments. *Indicates a statistically significant difference compared to control with p < 0.05.

**Figure 7:** Stable knockdown of miR-21 or STAT3 and overexpression of PDCD4 or catalase reduces the tumorigenicity of BEAS-2B cells chronic exposed to arsenic and injected into nude mice. Multiple sets of BEAS-2B cells were exposed to arsenic (0 or 0.5 μM) for 6 months: those stably silenced with either miR-21 or STAT3 shRNA, or transfected and overexpressing either PDCD4 or catalase, or the respective vector controls. Cells from different treatments were injected into the flanks of 6-week old athymic nude mice (2 × 10^6^ cells per mouse), and tumor volume was measured after 30 days. (**A**) Shown are the representative images of excised tumors and (**B**) graphic representation of tumor volume for each treatment group. (**C**) The relative miR-21 level was determined by Taqman real-time PCR. (**D**) PDCD4 protein expression was detected by immunohistochemistry. Results indicate that arsenic-induced tumorigenicity is associated with an increased levels of miR-21 and STAT3 while PDCD4 is decreased. Data presented in the bar graphs are the mean ± SD of three independent experiments. *^#^Indicates a statistically significant difference from respective control cells with p < 0.05.

**Figure 8:** Stable knockdown of miR-21 or STAT3 and overexpression of PDCD4 in AsT cells suppresses tumorigenesis. BEAS-2B cells were maintained in a medium containing arsenic (0.5 μM) for 6 months, and then cells were cultured in 0.35% soft agar for 5 weeks. (**A**) The arsenic-transformed cells (AsT) from anchorage-independent colonies were selected and maintained in DMEM. Passage-matched cells without arsenic treatment were used as the control. (**B**) The relative miR-21 level, determined by Taqman real-time PCR, was increased. (**C**) Total cell lysates were prepared for western blot analysis; apparent PDCD4 protein levels decreased. (**D–E**) Clonogenic assays were used to determine tumor cell proliferation. Cells (300) from indicated treatments were seeded into each of three dishes (60 mm diameter), and grown for an additional 10 days, then stained with crystal violet. Colony numbers in the entire dish were counted. (**D**) Images of representative plates for each treatment showing clonogenic activity, and (**E**) graphic representation of colony counts. Cells from indicated treatments were injected into the flanks of 6-week old athymic nude mice (2 × 10^6^ cells per mouse) and tumor volume was measured after 30 days. (**F**) Images of representative tumors excised from mice from each treatment group and (**G**) the associated tumor volumes were obtained. Knockdown of miR-21 or STAT3 and overexpression of PDCD4 inhibited tumor growth. (**H**) The relative miR-21 level for each treatment, determined by Taqman real-time PCR, was decreased relative to levels obtained from vector control tissues. (**I**) Representative images immunohistochemical staining show increased PDCD4 protein expression and (**J**) STAT3 phosphorylation. Data presented in the bar graphs are the mean ± SD of three independent experiments. *^#^Indicates a statistically significant difference from respective control cells with p < 0.05.

**Figure 9:** PDCD4 suppression by arsenic down-regulates E-cadherin and increases the accumulation of β-catenin and TCF4 in the nucleus. BEAS-2B cells were exposed to (**A**) acute (2.5, 5 and 10 μM arsenic for 24 h) and (**B**) chronic arsenic (0.1, 0.25 and 0.5 μM arsenic for 6 months) treatments. Total cell lysates were prepared for western blot analysis. Representative images of fluorescence immunostaining for (**C**) E-cadherin (**D**) β-catenin and (**E**) TCF4 of BEAS-2B cells with chronic arsenic treatment (0.5 μM). Arsenic treatment resulted in apparent increases for active-β-catenin and TCF-4, and decreases for E-cadherin protein levels.

**Figure 10:** PDCD4 suppression by arsenic stimulates β-catenin/TCF-dependent transcription of uPAR and c-Myc. BEAS-2B cells were exposed to various concentrations of arsenic (0.1, 0.25 and 0.5 μM) for 6 months. (**A**) Expression levels for c-Myc and uPAR, analyzed by western blot, showed apparent increases. To evaluate invasive capacity 1 × 10^5^ cells from each group were seeded on the top chamber of 24-well plate culture inserts coated with 20 μl of matrigel in duplicate. Cells were cultured for additional 48 h. Invaded cells on the bottom of insert were (**B**) stained and (**C**) quantified. (**D–E**) For the ChIP analysis, the TCF4 binding regions on uPAR and c-Myc promoters were identified. Chromatin isolated from BEAS-2B cells with chronic arsenic exposure were immunoprecipitated with an anti-TCF4 antibody or control mouse IgG. The TCF4 binding to the uPAR and c-Myc promoters was analyzed by RT PCR with specific primers. Arsenic increased the invasive capacity and binding of TCF4 complex to the uPAR and cMyc promoters. (**F**) Proposed mechanism of arsenic-induced malignant cell transformation and carcinogenesis. Data presented in the bar graphs are the mean ± SD of three independent experiments. *Indicates a statistically significant difference compared to control with p < 0.05.
